RETRACTED

# miRNA-448 Regulates the Development of Glioblastoma (GBM) by Regulating Rho-Associated Protein Kinase 1

**DOI:** 10.1155/2022/2502010

**Published:** 2022-03-03

**Authors:** Chang Liu, Bin Zhu, Meng Zhong, Jinsuo Bao

**Affiliations:** Neurosurgery Department, Affiliated Hospital of Inner Mongolia University for the Nationalities, Tongliao 028007, China

## Abstract

**Background:**

Glioblastoma (GBM) is an aggressive adult brain tumor that poses a huge threat to people's health. Previous studies have shown that microRNAs (miRNAs) are important regulators in the progression of GBM. However, the role of miR-448 in GBM remains largely unknown. Therefore, the regulatory mechanism of miR-448 in the development of GBM is elucidated in this study.

**Methods:**

The protein and mRNA expressions of miR-448 and ROCK1 were measured by Western blot analysis and RT-qPCR. Cell proliferation, migration, and invasion were detected by CCK-8 assay and Transwell assay. The relationship between miR-448 and ROCK1 was probed by luciferase reporter assay.

**Results:**

miR-448 expression was downregulated in GBM tissues and cells. And poor clinical outcomes of GBM patients were related to miR-448 downregulation. Functionally, overexpression of miR-448 restrained cell viability, migration, and invasion in GBM. Additionally, miR-448 reduced ROCK1 expression by binding to its 3′-UTR. Moreover, knockdown of ROCK1 inhibited the progression of GBM. Furthermore, overexpression of ROCK1 abolished the antitumor effect of miR-448 in GBM.

**Conclusion:**

miR-448 restrained cell viability, invasion, and migration in GBM by inhibiting ROCK1 expression.

## 1. Introduction

Glioblastoma (GBM) is a grade IV glioma, which mainly occurs in middle-aged people aged 40-60 years. The overall prognosis of GBM patients is poor [1]. Treatment of GBM is mainly neurosurgical resection, postoperative radiotherapy, and concurrent chemotherapy [2]. In general, the mean survival time of GBM patients after surgery, chemotherapy, and radiotherapy is approximately 14 months, and most GBM patients have a poor prognosis [3]. Today, targeted therapy and biological therapy have become the new direction of GBM treatment [4, 5] and also help to prolong the survival of patients. Therefore, exploring new therapeutic targets is of great significance for GBM patients.

It is well known that microRNAs (miRNAs) are involved in the regulation of cellular functions by negatively regulating target genes [6]. Moreover, increased miRNAs exhibit effects in GBM progression. miR-365 was downregulated and suppressed cell proliferation and migration by downregulating PAX6 in GBM [7]. Conversely, miR-374b was upregulated and promoted GBM progression by suppressing GATA3 [8]. These studies suggest that dysregulation of miRNAs is involved in the pathogenesis of GBM. Recently, the specific role of miR-448 has drawn our attention. For instance, downregulated miR-448 was found to alleviate spinal cord ischemia/reperfusion injury by upregulating SIRT1 [9]. In human ovarian and breast cancers, miR-448 expression was found to be reduced [10, 11]. Functionally, miR-448 restrained the invasion and proliferation of osteosarcoma cells [12]. In addition, miR-448 has been shown to play a critical role in suppressing pancreatic cancer [13]. However, the functional role of miR-448 in GBM has not been investigated in detail. Hence, this study is aimed at explaining the role of miR-448 in GBM.

RETRACTED

In previous studies, Rho-associated protein kinase 1 (ROCK1) has been reported to play a role in malignancies. Increased expression of ROCK1 has been detected in gastric cancer and osteosarcoma [14, 15]. Furthermore, ROCK1 has been shown to accelerate cell growth and motility in pancreatic and prostate cancers [16, 17]. Additionally, ROCK1 has been shown to be involved in tumorigenesis by interacting with miR-202 or miR-124 [18, 19]. Besides that, it has been suggested that ROCK1 mRNA has great diagnostic value in glioma patients [20]. And ROCK1 was found to promote glioma cell invasion [21]. However, the interaction between miR-448 and ROCK1 remains unclear in GBM. Therefore, this study involved some related experiments to demonstrate whether miR-448 plays a role in GBM by binding to ROCK1. Meanwhile, this study also explored how miR-448 regulates GBM progression. These findings will help to explain the molecular mechanism of miR-448 in the development of GBM.

## 2. Materials and Methods

### 2.1. Clinical Tissues

This study included 60 GBM patients from the Affiliated Hospital of Inner Mongolia University for the Nationalities. All patients signed the informed consent form and only underwent surgery. Our study was approved by the Institutional Ethics Committee of Affiliated Hospital of Inner Mongolia University for the Nationalities.

### 2.2. Cell Culture and Transfection

Primary normal human astrocytes (NHAs) and GBM cell lines A-172 MG, T98G were purchased from ATCC (Manassas, VA, USA). These cells were cultured in culture solution (90% DMEM+10% FBS), 5% CO_2_, and 37°C.

miR-448 mimics and inhibitor or ROCK1 overexpression plasmids and siRNA (RiboBio, Guangzhou, China) were transfected into A-172 MG cells using Lipofectamine 3000 (Invitrogen, Carlsbad, USA).

### 2.3. RNA Isolation and RT-qPCR

TRIzol reagent (Sigma, USA) was used for total RNA isolation. MicroRNA reverse transcription kit (Takara, Dalian, China) was used to reverse transcribe cDNA. RT-qPCR assay was performed by using SYBR Green Master Mix II (Takara). U6 and GAPDH are used as internal references. The relative expression of miR-448 and ROCK1 was calculated by the 2^−△△ct^ method. The primer sequences have been shown in Table 1.

RETRACTED

### 2.4. Transwell Assay

Cell invasion was detected using Matrigel. A-172 MG cells (4 × 10^3^ cells/well) were added to the upper chamber. DMEM medium (10% FBS) was added to the lower chamber to induce cell move. After 24 h incubation, the moving cells were stained with 0.1% crystal violet. With the exception of Matrigel, the steps of cell migration are the same as for invasion. Cell motility was observed with a light microscope.

### 2.5. CCK-8 Assay

A-172 MG cells (3 × 10^3^/well) were cultured in DMEM medium for 24, 48, 72, and 96 h. Then, 10 ml of CCK-8 (Dojindo, Kumamoto, Japan) was added to incubate the cells for 4 h. Finally, the optical density at 450 nm was measured by a microplate reader (Molecular Devices).

### 2.6. Dual Luciferase Reporter Assay

The pmirGLO luciferase reporter vector (Promega, USA) was inserted with Mut-ROCK1-3′UTR or Wt-ROCK1-3′UTR. Then, the luciferase vector was transfected into A-172 MG cells containing miR-448 mimics for 48 h. Luciferase activity was measured by dual luciferase assay system (Promega, USA).

### 2.7. Western Blot Analysis

RIPA buffer (Beyotime, Shanghai, China) was employed to lyse protein sample. Then, protein was separated by 10% SDS-PAGE. We transferred protein samples into PVDF membranes and blocked it with 5% nonfat milk. Then, protein was incubated overnight at 4°C with Bax (rabbit polyclonal antibody; dilution, 1 : 500; cat. no. 137321), Bcl-2 (rabbit polyclonal; dilution, 1 : 500; cat. no. ab45171), ROCK1 (rabbit polyclonal; dilution, 1 : 1,000; cat. no. ab196495), and GAPDH (rabbit monoclonal, dilution, 1 : 1,000; cat. no. ab181602) primary antibodies (Abcam, Shanghai, China). After washing, the protein was continued to be incubated with secondary antibodies (mouse antirabbit, dilution, 1 : 2,000; cat. no. 58802; Abcam) for 1 h. Finally, protein bands were assessed by ECL kit (Beyotime). Quantity One 4.52 analysis software was used to measure the gray value of the bands. The relative expression of the target protein (IOD) = the gray value of the target protein/the gray value of the internal reference GAPDH.

### 2.8. Statistical Analysis

Data were analyzed by SPSS 17.0 and shown as mean ± SD. Figures were made with Graphpad Prism 6. Student's *t*-test, Chi-squared test, and ANOVA with Turkey's multiple comparison tests were used to calculate differences. *P* < 0.05 indicates a significant difference.

RETRACTED

## 3. Results

### 3.1. miR-448 Was Downregulated in GBM

First, the expression of miR-488 was found to be lower in GBM tissues than in normal tissues (*P* < 0.01, Figure 1(a)). Compared with NHAs cells, miR-448 was also downregulated in A-172MG and T98G cells (*P* < 0.01, Figure 1(b)). Meanwhile, the histological grade of glioma patients was associated with dysregulation of miR-448 (Table 2; *P* < 0.05), suggesting that dysregulation of miR-448 indeed exists in GBM development. Then, we found that miR-448 mimics increased its expression, while miR-448 inhibitor decreased its expression in A-172MG cells (*P* < 0.01, Figure 1(c)).

### 3.2. Overexpression of miR-448 Restrained GBM Progression

Next, overexpression of miR-448 was found to inhibit cell proliferation, whereas downregulation of miR-448 accelerated A-172MG cell proliferation (*P* < 0.01, Figure 2(a)). As shown in Figure 2(b), miR-448 mimics promoted Bax expression and reduced Bcl-2 expression. Correspondingly, downregulation of miR-448 inhibited Bax expression and promoted Bcl-2 expression (Figure 2(b)). Cell migration was found to be inhibited by miR-448 mimics and promoted by miR-448 inhibitor (*P* < 0.01, Figure 2(c)). In addition, the same effect of miR-448 on A-172MG cell invasion was also identified (*P* < 0.01, Figure 2(d)). Overall, overexpression of miR-448 restrains cell viability, migration, and invasion in GBM.

### 3.3. miR-448 Directly Targets ROCK1

Furthermore, the TargetScan database (http://www.targetscan.org/) showed that miR-448 can bind to ROCK1 (Figure 3(a)). Next, a luciferase reporter assay showed that the miR-448 mimics reduced Wt-ROCK1 luciferase activity (*P* < 0.01, Figure 3(b)). In addition, ROCK1 expression was inhibited by miR-448 upregulation and promoted by miR-448 downregulation in A-172MG cells (*P* < 0.01, Figure 3(c)). Compared to normal tissues, ROCK1 was upregulated in GBM tissues (*P* < 0.01, Figure 3(d)). Meanwhile, miR-448 was also found to negatively regulate ROCK1 expression in GBM tissues (*P* < 0.01, *R*^2^ = 0.7078; Figure 3(e)). The above results suggest that miR-448 reduces ROCK1 expression by binding to its 3′-UTR.

### 3.4. Knockdown of ROCK1 Impeded the Progression of GBM

Next, the dysregulation of ROCK1 was detected in GBM. We found that the expression of ROCK1 was higher in A-172MG and T98G cells than in NHAs cells (*P* < 0.01, Figure 4(a)). Then, A-172MG cells with ROCK1 siRNA were prepared to explore the role of ROCK1 in GBM. ROCK1 was found to be downregulated by its siRNA (*P* < 0.01, Figure 4(b)). Furthermore, ROCK1 knockdown inhibited cell proliferation in A-172MG cells (*P* < 0.01, Figure 4(c)). ROCK1 silencing enhanced Bax expression and decreased Bcl-2 expression in A-172MG cells (*P* < 0.01, Figure 4(d)). In addition, ROCK1 silencing suppressed cell migration and invasion (*P* < 0.01, Figures 4(e) and 4(f)). Combined with these results, ROCK1 is considered to be an oncogene in GBM.

RETRACTED

### 3.5. Upregulation of ROCK1 Abolished the Suppressive Role of miR-448 in GBM

A-172MG cells with miR-448 mimics and ROCK1 vector were used to confirm the interaction of miR-448 and ROCK1 in GBM. ROCK1 vector restored the downregulation of ROCK1 induced by miR-448 mimics (Figure 5(a)). More importantly, miR-448 mimic-mediated inhibition of cell proliferation was impaired by upregulation of ROCK1 (Figure 5(b)). The reversal effect of ROCK1 on Bcl-2/Bax expression was also found in A-172MG cells (Figure 5(c)). Meanwhile, upregulation of ROCK1 attenuated the inhibitory effect of miR-448 on A-172MG cell migration and invasion (Figures 5(d) and 5(e)). Briefly, upregulation of ROCK1 restrains the antitumor effect of miR-448 in GBM.

## 4. Discussion

Recently, an increasing number of miRNAs are found to play carcinogenic or anticancer role in GBM. For example, miR-1225-5p has been reported to be downregulated and act as a tumor inhibitor in GBM by targeting IRS1 [22]. Nonetheless, the regulatory mechanism of miR-448 in GBM has not been reported in previous studies. In this study, miR-448 was found to be downregulated and exert inhibitory effect in GBM. Specifically, we also found that downregulation of miR-448 was associated with histological grade of GBM patients. Our results also showed that upregulation of miR-448 inhibited cell viability, migration, and invasion in GBM. At the same time, upregulation of miR-448 induced apoptosis in GBM by reducing Bcl-2 expression and promoting Bax expression. To go much further, miR-448 suppressed ROCK1 expression by binding to its 3′-UTR. Moreover, upregulation of ROCK1 abolished the antitumor effect of miR-448 in GBM. Taken together, our findings reveal that miR-448 acts as a tumor suppressor in GBM through binding to ROCK1.

Recently, downregulation of miR-448 expression has been observed to be reduced in osteosarcoma and breast cancer [23, 24], which is consistent with our results. Additionally, low miR-448 expression has been reported to be associated with advanced tumor stage and metastasis in hepatocellular carcinoma [25]. Similarly, poor clinical outcomes in GBM patients were also found to be associated with downregulation of miR-448. Functionally, miR-448 inhibited the invasion and proliferation of gastric cancer cells by controlling ADAM10 [26]. Additionally, it was shown that miR-448 induced suppression of ovarian cancer cell metastasis by inhibiting CXCL2 [11]. These studies are consistent with our results. In addition to this, miR-448 was found to affect cell viability by regulating Bax/Bcl-2 in GBM. miR-448 exhibited effect in human cancers by mediating the expression of some genes such as IGF1R [27]. Here, miR-448 was found to be involved in GBM progression by interacting with ROCK1.

RETRACTED

ROCK1, an oncogenic factor, has been found to be upregulated in osteosarcoma and colorectal cancer [28, 29]. Here, upregulation of ROCK1 was also detected in GBM. ROCK1 silencing was shown to inhibit the invasion, migration, and proliferation of laryngeal squamous cell carcinoma cells [30]. The present study also showed that ROCK1 has an oncogenic role in GBM, which is similar to previous studies. Moreover, miR-145 has been found to inhibit cell proliferation and promote apoptosis in hepatocellular carcinoma by downregulating ROCK1 [31]. miR-101 suppressed the invasion, migration, and proliferation of osteosarcoma cells by downregulating ROCK1 [32]. In our study, miR-448 was found to hinder the development of GBM by regulating ROCK1. All these findings suggest that the miR-448/ROCK1 axis is involved in GBM progression by inhibiting cell viability, invasion, and migration.

## 5. Conclusion

In conclusion, decreased miR-448 expression in GBM is associated with poor clinical outcomes. Furthermore, miR-448 restrains GBM progression by downregulating ROCK1. Although we have explained partial functions of miR-448 in GBM, the specific regulatory network of miR-448 needs to be explained in GBM.

## Figures and Tables

**Figure 1:** miR-448 was downregulated in GBM. (a) The mRNA miR-448 expression in GBM tissues. (b) The miR-448 expression in A-172MG, T98G, and NHAs cells. (c) miR-448 expression was examined in A-172MG cells with its mimics or inhibitor. ∗∗*P* < 0.01.

**Figure 2:** Overexpression of miR-448 restrained GBM progression. (a) miR-448 regulated cell proliferation in A-172MG cells. (b) miR-448 regulated protein expressions of Bax and Bcl-2 in A-172MG cells. (c, d) Cell migration and invasion were measured in A-172MG cells with miR-448 mimics or inhibitor. ∗*P* < 0.05, ∗∗*P* < 0.01.

**Figure 3:** miR-448 directly targets ROCK1. (a) The binding sites between ROCK1 and miR-448. (b) Luciferase reporter assay. (c) miR-448 regulated ROCK1 expression. (d) ROCK1 expression in GBM tissues. (e) miR-448 was negatively correlated with ROCK1 in GBM tissues. ∗∗*P* < 0.01.

**Figure 4:** Knockdown of ROCK1 impeded the progression of GBM. (a) ROCK1 expression was measured in A-172MG, T98G, and NHAs cells. (b) ROCK1 expression was measured in A-172MG cells with its siRNA. (c) Cell proliferation in A-172MG cells with ROCK1 siRNA. (d) ROCK1 regulated protein expressions of Bax and Bcl-2 in A-172MG cells. (e, f) Cell migration and invasion in A-172MG cells with ROCK1 siRNA ∗∗*P* < 0.01.

RETRACTED

**Figure 5:** Upregulation of ROCK1 abolished the inhibitory effect of miR-448 in GBM. (a) The expression of ROCK1 in A-172MG cells containing miR-448 mimics and ROCK1 vector. (b) Cell proliferation in A-172MG cells containing miR-448 mimics and ROCK1 vector. (c) Bax and Bcl-2 in A-172MG cells containing miR-448 mimics and ROCK1 vector. (d, e) Cell migration and invasion in A-172MG cells containing miR-448 mimics and ROCK1 vector *r*∗∗*P* < 0.01.

**Table 1:** The primers for RT-qPCR.

Primers		
miR-448	5′-TTGCATATGTAGGATGTCCCAT-3′	5′-CTCAACTGGTGTCGTGGGGCCA-3′
ROCK1	5′-GGTGGTCGGTTGGGGTATTT-3′	5′-AACTGGTGCTACAGTGTCTCG-3′
U6	5′-CGCTTCGGCAGCACATATAC-3′	5′-TTCACGAATTTGCGTGTCAT-3′
GAPDH	5′-GGTGAAGGTCGGAGTCAACG-3′	5′-CAAAGTTGTCATGGATGHACC-3′

**Table 2:** Relationship between miR-448 expression and their clinic-pathological characteristics of glioma patients.

Characteristics	Cases	miR-448		*P* value
		High	Low	
Age (years)				0.21
≥55	34	10	24	
<55	26	7	19	
Gender				0.38
Male	36	12	24	
Female	24	5	19	
Tumor size (mm)				0.31
≤5.0	12	6	6	
>5.0	48	11	37	
WHO grade				0.02∗
I-II	10	5	5	
III-IV	50	12	38	

WHO: World Health Organization; statistical analyses were performed by the *χ*^2^ test. ∗*P* < 0.05 was considered significant.

## Data Availability

Data to support the findings of this study is available on reasonable request from the corresponding author.
